# Analysis of Data on Fludarabine, Cyclophosphamide, and Rituximab Chemoimmunotherapy for Chronic Lymphocytic Leukemia Shows High Patient Heterogeneity and the Need for More Consideration of Individualized Treatment

**DOI:** 10.1155/2022/7451395

**Published:** 2022-10-03

**Authors:** Xiaoli Xu, Ying Zhao, Haiyan Ye, Yonglei Qi, Wenning Xu, Yiwen Ling, Shaojiang Yang

**Affiliations:** Department of Hematology, First People's Hospital of Foshan, Foshan, China

## Abstract

**Methods:**

Data from single-cell RNA sequencing (RNA-seq) of CLL patients were obtained from the Gene Expression Omnibus database. The R package was utilized to analyze the data, and the relation of results was predicted via the GeneMANIA website. The information of 7 samples covered three stages: observation stage, pretreatment by CIT with rituximab, fludarabine, and cyclophosphamide (pre-CIT), and post-CIT. The differentially expressed genes (DEGs) were identified, and functional enrichment analyses were performed. B cell subpopulations and pseudotime trajectories analysis was conducted.

**Results:**

A total of 70,659 DEGs were identified. Each patient's DEGs presented their own characteristics, with low similarity. Therefore, it is difficult to identify potential hub genes. Similarly, pathway enrichment analysis showed significant tumor heterogeneity among CLL patients. Analysis of relapsed post-CIT compared to the observation stage suggested that the *TP53* pathway should be taken seriously as it is closely related to treatment strategy and patient prognosis.

**Conclusions:**

Tumor heterogeneity may be a more common manifestation of CLL. Individualized treatment should be considered for CLL. *TP53* abnormality and its regulatory factors should still be the focus of CLL diagnosis and treatment.

## 1. Introduction

Chronic lymphocytic leukemia (CLL) is one of the most common adult leukemia in the world. The incidence of CLL is estimated to be more than 4-6 per 100,000 population annually in developed countries, and the ratio of men to women is about 2 : 1 [1, 2]. Although the median age at diagnosis is 72 years, 10% of CLL patients are younger than 55 years [3]. Diagnosis as early as possible may help improve patient prognosis. Currently, clinical diagnostic criteria are based on the number and morphology of monoclonal B lymphocytes. The number of monoclonal B lymphocytes is over 5 x 10/L in the peripheral blood [3]. Meanwhile, the characteristic of most leukemia cells found in the blood smear is small and mature-appearing lymphocytes. The cells present a narrow border of cytoplasm, a dense nucleus lacking discernible nucleoli and partially aggregated chromatin [3]. In terms of cellular molecules, several B cell surface antigens are coexpressed, such as CD19, CD20, and together with CD5, CD23, CD43, and CD200 [4]. Although it can be clearly diagnosed as CLL based on the clinical diagnostic criteria and markers of the cell surface, there is indeed still a great deal of uncertainty in the progression and prognosis of the tumor. It has been identified that CLL presents an inherited genetic susceptibility, the family members of CLL patients with 6-9 folds increased risk [3]. This has led to the exploration of the deeper molecular mechanisms characterizing CLL in order to achieve precise diagnosis and treatment.

In general practice, treatment of CLL relies on the Rai and Binet staging systems and the presence of symptoms [5, 6]. Most patients of early-stage (Rai 0; Binet A) present with asymptomatic and should be monitored without therapy, that is the observation stage. Patients with advanced (Rai III and IV; Binet B, and C) symptomatic disease and rapidly progressive lymphocytosis usually need to be treated and could benefit from treatment [1, 3, 7]. Chemoimmunotherapy (CIT) using the anti-CD20 monoclonal antibody rituximab and fludarabine plus cyclophosphamide (FCR) has become the standard treatment for most CLL patients [1]. However, recent developments in the diagnosis and treatment of CLL have emphasized individualized treatment strategies. It is recommended that the therapy decision is based on the integration of the factors related to the neoplasm and the factors related to the patient [2]. Treatment of CLL patients should take into account their disease subsets, treatment tolerance factors such as age, comorbidities, and genetic factors such as *TP53* mutation/deletion [2]. Therefore, in addition to consideration of different clinical stages, the patient's chromosomal or genetic abnormalities should also be referred to. The implementation of appropriate anticancer treatment on this basis may help improve prognosis. However, the molecular pathological mechanism of CLL is complex and has individual characteristics. Even an excellent model needs frequent updating and tailoring to a particular population of CLL patients to sustain its predictive effectiveness [8]. This requires extensive in-depth molecular mechanistic exploration work, including research methods and strategies.

With the development of next-generation sequencing technology, bioinformatics analysis brings a more comprehensive and novel perspective to decode life mysteries, detect pathogens, and improve quality of life [9]. Whole-genome and -exome sequencing has contributed to the characterization of the mutational spectrum of the disease. Sequencing analysis studies on CLL are gradually being reported. A previous study of RNA-sequencing (RNA-seq) in different subpopulations of normal B lymphocytes and CLL cells has shown differential expression of transcriptional elements, including genes of protein-coding, noncoding RNAs, and pseudogenes [10]. Differentially expressed genes (DEGs) between B cells and CLL specimens were revealed [10, 11]. In addition, there were studies around small noncoding RNAs (sncRNAs), subtype-specific epigenome signatures, and transcription regulatory networks of CLL [12, 13]. In the area of drug tolerance, Landau et al. suggested that the frequently observed clonal shifts during the early treatment period of CLL, heralded the emergence of drug-resistant clones [14]. However, few studies have been reported on bioinformatics analysis of CLL treatment and relapse in recent years.

This research has explored the genetic characteristics and differences in signaling pathway activity among CLL patients and pre- and post-CIT treatment based on data analysis. The initial goal was to uncover genes and signaling pathways that may play a critical role in CLL treatment and prognosis. However, the findings suggested that the heterogeneity among patients with CLL and at different stages of the disease was evident. When considering genetic abnormalities that are closely related to CLL, such as the *TP53* pathway, individualized patient care should also be taken into account.

## 2. Materials and Methods

### 2.1. Data

Single-cell RNA sequencing data of GSE165087 were obtained from Gene Expression Omnibus (GEO) datasets (https://www.ncbi.nlm.nih.gov/geo/query/acc.cgi?acc=GSE165087). The information of patient 1, patient 2, and patient 3 was chosen, including 10 samples that cover three stages. They are observation (OB) (CLL 1_1.1, CLL 1_1.2), pretreatment by CIT with fludarabine, cyclophosphamide and rituximab (pre-CIT) (CLL 1_3.1, CLL 1_3.2, CLL 2_1, CLL 3_1), and post-treatment by CIT (post-CIT) (CLL 1_5.1, CLL 1_5.2, CLL 2_2, CLL 3_2). We combined the two technical repetitions into one to optimize the structure. As a consequence, we reorganized 7 samples (CLL 1-1, CLL 1-2, CLL 1-3, CLL 2-1, CLL 2-2, CLL 3-1, and CLL 3-2) to further analyze. The analysis process of this study is shown in Figure 1.

### 2.2. Quality Control, Dimensionality Reduction, and Data Integration

The single-cell RNA-seq data were imported into the Scater package (version 1.14.6) [15]. The median absolute deviation (MAD) was used to judge the unique molecular identifiers (UMI) and feature count outliers. We used the function of Outlier to remove cells with a log-library size of more than 3 MADs (the median log-library size) and cells with a mitochondrial gene expression ratio greater than 20% which usually corresponds to dead or injured cells. To eliminate differences in gene expression between cells based on count data, the global scaling normalization method LogNormalize was applied to standardize the measurement of the characteristic expression for each cell with the total expression. And then 2000 genes with high variation were extracted by the VST method, based on a large coefficient of variation. After integrating multiple samples with the function of IntegrateData, we scaled the data by linear transformations to ensure each gene was given the same weight with a mean of 0 and a variance of 1. For the sake of reducing the computational burden and the noise in the data, principal component analysis (PCA) was used for preliminary dimensionality reduction. We used the Seurat package (version 3.1.4) function of FindNeighbors and FindClusters to cluster the cells [16]. The clustering data were projected into low-dimensional space via uniform manifold approximation and projection (UMAP), a nonlinear dimension reduction technique retaining the original topological structure.

### 2.3. Cell Annotation and Ratio Calculation

Following obtaining 8 stable cell subpopulations from cluster analysis, we used the function of the FindAllMarkers Wilcoxon rank-sum test to determine the multiple gene differences between the cell group and other groups with the average value of avg_logFC. Database PanglaoDB and CellMarker provided marker genes in different cell types and the SingleR algorithm [17] assisted the verification of identified cell types by calculating the Spearman correlation between the expression profile of each cell and that of each reference sample so that the 6 types of cell subpopulations were determined. In the present study, we analyzed B cells.

### 2.4. Variance Analysis and Pathway Enrichment

The gene expression variance evaluation of B cells was conducted by R package, which was compared in each group via Kruskal-Wallis Test. Gene Set Enrichment Analysis (GSEA) was implemented in the Fgsea package (version 1.12.0) to determine pathways [18]. Sequencing was performed according to LogFC of rank-sum test difference analysis as the sorted gene list. Further GSEA analysis was performed via the Kyoto Encyclopedia of Genes and Genomes (KEGG) gene set. Gene Set Variation Analysis (GSVA) package (version 1.34.0) [19] and the subsequent analysis described by MSigDB databases were driven to pathways of Geno Ontology (GO) annotation, hallmarker terms, and KEGG. As a footnote, GO and KEGG analyses were used to estimate the functions of DEGs, concluding with the biological process (BP), cell composition (CC), and molecular function (MF), which were analyzed by Fisher's test. *P* < 0.05 was regarded as statistically significant.

### 2.5. Gene Association Network

We chose differentially expressed genes interested and differentially enrichen pathway interested and performed the latent relation among them via GeneMANIA (http://genemania.org/), including physical interactions, coexpression, colocalization, genetic interaction, and pathway.

### 2.6. B Cell Subpopulations Clustering

To explore the pathways and functions involved in each subpopulation of B cells, gene enrichment analysis was performed for each subpopulation. Rank-sum test was used to compare the differences in gene expression levels of B cell subsets.

### 2.7. B Cell Pseudotime Trajectories Analysis

Pseudotime trajectories analysis refers to the construction of cell lineage development based on the changes in gene expression levels of different cell subpopulations over time which is a virtual time sequence according to the track of transformation and succession from cell to cell. Monocle uses an algorithm to learn the sequence of changes in gene expression that each cell must undergo as part of a dynamic biological process. Once it understands the overall trajectory of changes in gene expression, Monocle can place each cell in the right place within the trajectory. Monocle relies on a machine-learning technique called reverse graph embedding to construct single-cell trajectories. We used Monocle 2 package (v2.8.0) [20] to analyze cell state transitions and then we put the top 100 differentially expressed genes in the Seurat package to establish the pseudotime trajectories. The B cells state conducted origin of the pseudotime as orderCells. The abnormal gene expression profiles were set to root_state argument, and then we invoked orderCells, DDRTree reducing dimensions, and the plot_cell_trajectory plotting the minimum spanning tree. The top 100 differentially expressed genes of B cells were calculated by the function differential GeneTest. We performed genes meeting the thresholds with mean_expression ≥ 0.5 and dispersion_empirical ≥ 1∗ dispersion_ fit to present cells in pseudotime order.

### 2.8. Gene Variance Pseudotime Trajectories

Genes with similar trends were grouped into two categories. In one group, the expression was from low to high. We set the low state at the beginning of differentiation, and it decreased gradually with the increase of pseudotime. In the other group, the expression level was high at the beginning of differentiation and decreased gradually with the increase of pseudotime.

### 2.9. Statistical Analysis

All statistical analyses were carried out via the R package (http://www.r-project.org). A two-sided paired or unpaired Student's *t*-test and unpaired Wilcoxon rank-sum test were used for indication. *P* < 0.05 was considered to manifest statistical significance.

## 3. Results

### 3.1. Identification of DEGs in B Lymphocytes of CLL Patients

In the present study, 7 data series which covered 3 stages were analyzed. A total of 70,659 DEGs were identified. In order to screen the representative DEGs between pre-CIT and relapsed post-CIT in CLL patients, we took the top 20 genes with the largest expression in each group to draw a heat map according to logFC, as shown in (Figure 2(a)). However, the DEGs of patients lack commonalities, and each patient appeared to present his/her own characteristics (Figures 2(b)–2(d)). None of the high expression genes coincide among the three patients when comparing pre-CIT with relapsed post-CIT. There was only one gene, *JUN* (Jun proto-oncogene, AP-1 transcription factor subunit), with high expression in both patient 1 and 2, while other 5 genes including *CD47*, *HLA-DPA1*, *FCER2*, *CD79A*, and *IGLV2-14* were highly expressed in both patient 2 and 3 in the compared pre-CIT with post-CIT. But most encoded proteins of these genes were B cell antigen or involved in immune response, which did not reveal the underlying pathological mechanism of CLL very well. Similarly, none of the high expression genes coincide among the three patients compared relapsed post-CIT with pre-CIT. In the relapsed post-CIT, there were 2 genes, *TXNIP* and *EMP3*, presented high expression in both patient 1 and 2. 2 genes, *HLA-A* and *HLA-C*, presented high expression in both patient 1 and 3. And 3 genes, *ZFP36L2*, *HERPUD1*, and *ZFP36*, presented high expression in both patient 2 and 3. In addition to this, 17-19 of the 20 DEGs were not the same among patients, even the expression trends of some genes were reversed in different patients. Therefore, the results suggested that the DEGs of relapsed post-CIT presented significant heterogeneity among CLL patients.

The top 100 DEGs of each CLL patient were selected for pseudotime analysis and genes with similar trends were grouped together. The heat maps show clusters of genes with the same expression pattern (Figures 3(a)–3(c)). Similarly, the results also showed that the DEGs of pseudotime were heterogeneous among patients.

### 3.2. Pathway Enrichment Analyses of the Common DEGs of CLL Patients

To further explore the potential role of signaling pathways in the disease mechanism of CLL, we conducted pathway enrichment analysis across different stages of each patient according to DEGs. However, we found significant differences among CLL patients, suggesting significant heterogeneity (Figure 4). There were 5 pathways with the most significant differences of patient 1 which were the regulation of autophagy, ubiquitin-mediated proteolysis, and *TP53* signaling pathway, etc. (Figure 4(a)). Pathways with significant differences between pre-CIT and post-CIT in patient 2 were related to energy metabolism, these were glycosaminoglycan degradation, immune disorders, and the *TP53* signaling pathway, *etc.* (Figure 4(b)). Although it was somewhat similar between patient 3 and patient 2, more than half of the differential pathways were not consistent (Figure 3(c)). This result probably suggested that changes in energy metabolism and immune factors may affect the therapeutic efficacy of CLL, thereby affecting disease progression. However, there were individual differences in signaling pathway characteristics of different patients. No convincing molecular mechanism for CLL disease progression can be deduced yet from the results of the current pathway enrichment analysis. To further search for target pathways, we narrowed the scope and drew a network map of several major pathways that may be involved in CLL pathophysiology and their closely related genes for further analysis of potential targets (Figure 5). Among these, the *TP53* pathway and ubiquitin-mediated proteolysis pathway were closely related to the cell cycle process through multigene groups. This suggested that classical signaling pathways such as *TP53* may still be the main therapeutic entry point.

### 3.3. KEGG, Hallmark, and GO Pathway Enrichment Analyses of Patient 1

Heterogeneity of DEGs and pathways among patients suggested that it was better to perform individual analyses independently. To uncover the molecular metabolic characteristics of stability and progression of CLL, we further analyzed the differences between the observation stage and relapsed post-CIT in patient 1 (Figure 6). As shown in the KEGG graph analyzed by GSVA (Figure 6(a)), pathways with significantly increased activity in relapsed post-CIT compared to the observation stage were the *TP53* signaling pathway, ubiquitin-mediated proteolysis, immune abnormality, etc. (Figure 4(a)). Pathways with decreased activity were TGF-beta signaling pathway, other glycan degradation, hedgehog signaling pathway, etc. (Figure 6(a)). Hallmarks is a gene set related to tumor growth and metastasis dissemination, which helps to define the character of malignancies. Results of hallmark showed that pathways with significantly increased activity were the *TP53* signaling pathway, TNF*α* signaling via NFkB, apoptosis, etc. (Figure 6(b)). Pathways with decreased activity were energy metabolism and oxidative regulation, etc. (Figure 6(b)). There were a small number of resemblances between the observation stage and post-CIT containing the *TP53* pathway, which was in accordance with the result of KEGG. During the observation stage, the activity of the *TP53* pathway stayed low and started negative growth at the stage of pre-CIT and reversing to positive growth when post-CIT (Figure 6(b)). However, the results of GO showed that the organelle structure and function may vary at different stages of CLL progression (Figure 6(c)). These pathway enrichment analysis results from different focuses suggested that there were significant differences in the activities of pathways in the observation stage and the relapsed post-CIT, especially the *TP53* signaling pathway and energy metabolism pathway, which were closely related to malignant tumors.

### 3.4. B Cell Pseudotime Trajectories and DEGs of Subpopulations of Patient 1

The B cells lineage development was constructed as a pseudotime tree trajectory (Figure 7(a)), in which dots represented cells and cells with a similar situation were clustered together. We sorted out clusters of different stages of CLL in patient 1 (Figure 7(b)) and separated each state of the 3 stages (Figure 7(c)). The B cell pseudotime trajectories showed the virtual developmental model of the post-CIT was different from the observation stage. To better understand how treatment with CIT impacted B cells of CLL patients, we presented B cell subpopulations of each stage of patient 1 (Figure 7(d)). Although the B cell subpopulation clusters of different stages did not present significant differences, there was no similarity in DEGs between different B cell subpopulations and stages of B cells (Figures 7(e) and 7(f)). This suggested that subpopulations of B cells in the same patient also exhibited heterogeneity as CLL progresses.

## 4. Discussion

Exploring the pathological mechanism of CLL contributes to the update of its treatment strategy, but only a limited number of its pathogenesis and risk factors have been identified until now. There is still a long way to go to build accurate prognostic prediction models for CLL that can be effectively translated into the clinic [8]. CLL is one of the strongest inherited predispositions of hematological malignancies [1, 21, 22]. Intricate genetic factors bring challenges to the exploration of molecular mechanisms of CLL. Microarray technology such as RNA-seq may help us understand the significant differences in the molecular mechanisms between pre-CIT and post-CIT of CLL. However, the results of the present study showed significant heterogeneity among the patients and different stages of CLL. Furthermore, we focused on the differences between the steady stage of observation of CLL and the relapse after CIT treatment. Several well-known signaling pathways and genes such as *TP53* may be the potential target associated with disease progression and treatment. Individualized treatment strategies should be increasingly applicable to CLL patients.

Cancer is a disease which is dynamic and generally becomes more heterogeneous during the evolution course, which provides the fuel for resistance to treatment [23]. Tumor heterogeneity can be broadly divided into intertumoral and intratumoral heterogeneity. A recent study showed that around 95.1% of informative samples of cancer (2,658 cancer samples contained 38 cancer types) presented evidence of distinct subclonal expansions and frequent branching relationships between each other [24]. This indicated that tumor heterogeneity is pervasive. Single-cell RNA-seq analysis results of the present study showed significant differences in gene expression traits and active pathways among CLL patients, including pre-CIT and post-CIT, showing heterogeneity. Moreover, all these patients relapsed after CIT, and at the same time, heterogeneity predicts challenges for subsequent treatment and prognosis. Research on cancer brings us awareness that it is not a fixed course when cancer develops and progresses, maybe as an integrated destabilization of key cellular processes [23]. Cancer is dynamic and continues to evolve, which might ultimately generate a bulk tumor which is molecularly heterogeneous, the differential sensitivity levels to anticancer therapies are shown by distinct molecular signatures [23]. This probably pointed out one of the main reasons for the treatment bottleneck of cancer, including CLL, especially when it progresses from observation stage to relapsed post-CIT as this study showed. Previous studies of whole-exome sequencing of more than 1,000 CLL specimens and whole-genome sequencing of 200 CLL patients have revealed the presence of 0.9 mutations per megabase and a load of 10-30 nonsilent events per patient [14, 25–28]. Additionally, CLL is genetically heterogeneous, containing multiple clonal and subclonal populations [25]. The treatment tolerance and the abundance and identity of the selected subclones with their evolution were affected by the interactions of these subclones along with their response to internal or external constraint [25, 26, 28]. With exposure to sequential treatment, the genomic complexity of a tumor generally increases. Clonal evolution arises more frequently in tumors receiving CIT [28]. Although tumor heterogeneity poses challenges for treatment and prognosis, studying heterogeneity has fueled a shift in the treatment paradigm towards the use of personalized or genotype­guided approaches. Evidence has indicated that heterogeneity can predict resistance to both chemotherapies and targeted therapy and can inform prognostication, therefore, the assessment of tumor heterogeneity is essential for the development of effective treatment [23, 25, 29].

Although realizing that CLL is highly heterogeneous, the present study compared DEGs and signaling pathway activity between the observation stage and relapsed post-CIT of CLL to unearth potential factors which may affect CLL progression and treatment tolerance. Results showed that several well-known signaling pathways presented significant differences between CLL stabilization and progression, such as the *TP53* pathway. A previous study had identified that *TP53* aberrations predict an aggressive disease course and refractoriness to CIT [1]. Results of a randomized prospective trial (followed-up of 52.8 months) showed that *TP53* mutations in 8.5% of CLL patients and none of the patients with *TP53* mutation achieved a complete response [30]. A meta-analysis of an international consortium created an international prognostic index for CLL that integrated the major prognostic parameters [31]. *TP53* status (no abnormalities vs. del [17p] or *TP53* mutation or both) is one of the 5 independent prognostic factors [31]. *TP53* mutation was the strongest prognostic marker regarding progression-free survival (PFS) according to the multivariate analysis [30]. The median PFS and overall survival (OS) of patients with *TP53* mutation were significantly decreased compared with patients without *TP53* mutation. The prognostic implication of *TP53* dysregulation is related to its association with resistance to DNA damaging agents and a decreased time to first treatment and unfavorable OS [32–34]. Accordingly, *TP53* inactivation is one of a major determinants of therapeutic decisions [25]. Patients with a *TP53* mutation or del (17p) are in a high-risk category and should be treated with targeted agents [35]. An allogeneic hematopoietic stem cell transplantation (SCT) may be considered in relapsing patients with *TP53* mutations or del (17p), or patients that are refractory to inhibitor therapy [35]. However, some patients do not have suitable access to SCT. It is still recommended that the presence of del17p and *TP53* disruptions should be tested for patients of treatment-naive requiring therapy [25]. If these lesions are present, even at the subclonal, treatment of genotoxic drugs (alkylating agents, anthracyclines, or purine analogues) should not be performed, for a poor response to genetic lesions will hamper DNA repair [26, 36, 37]. An earlier study had shown that the median PFS of CLL patients with *TP53* abnormalities treated using FCR or other CIT combinations was less than 18 months [34]. Thus, ibrutinib and venetoclax are recommended for patients with *TP53* mutations upfront treatment, for the estimated median PFS of more than 30 months [38–40]. For CLL patients with relapsed or refractory after CIT treatment, targeted therapies may be the best option [25]. Results of a recent clinical trial showed that the 5-year PFS rate of patients receiving ibrutinib was 92% in treatment-naive patients and 44% in relapsed or refractory patients, the median PFS was 51 months in heavily pretreated patients receiving ibrutinib [41]. Taking this into account, the combination of venetoclax and rituximab was approved in 2018 by the FDA, and it is an option worth considering for the treatment of relapsed or refractory CLL [42]. Although these studies have brought new insights into CLL, new breakthroughs are still needed in individualized treatment and prognosis. The signaling pathways and their regulators related to CLL progression still need to be further studied to bring novel ideas for individualized treatment decisions.

The present study still has certain limitations. The limited number of samples for different stages of CLL and CIT treatment may cause bias in the analysis of existing data. This study has not yet conducted experimental verification of the current inferences and hypothesis, especially key gene expression and signaling pathways. The new discoveries and viewpoints of the results of this study need to be proved by future experiments.

## 5. Conclusion

In conclusion, tumor heterogeneity may be a more common manifestation of CLL. Given this, in-depth diagnosis and individualized treatment strategies may be required for CLL management. Among these, *TP53* abnormality and its regulatory factors should still be the focus of CLL diagnosis and treatment.

## Figures and Tables

**Figure 1:** The analysis process.

**Figure 2:** DEGs in B lymphocytes of CLL patients. (a) The top 20 genes with the largest expression in each group. (b) The DEGs of patient 1, compared between observation stage and post-CIT. (c) The DEGs of patient 1, compared between pre-CIT and post-CIT. (d, e) The DEGs of patient 2 and 3, compared between pre-CIT and post-CIT.

**Figure 3:** The top 100 DEGs pseudotime heat map of the three CLL patients.

**Figure 4:** Pathway enrichment analyses of the common DEGs of CLL patients. (a) Patient 1, (b) patient 2, and (c) patient 3.

**Figure 5:** Pathway network.

**Figure 6:** KEGG, Hallmark, and GO pathway enrichment analyses of patient 1. (a) KEGG, (b) Hallmark, and (c) GO.

**Figure 7:** B cell pseudotime trajectories and DEGs of subpopulations of patient 1. (a) The colors of B cells lineage development darkened with the pseudotime developing. (b) The colors of B cells lineage development darkened with the WBC increasing.(c) The B cell pseudotime trajectories were distinguished to 3 stages of CLL. (d) The B cell pseudotime trajectories of each stage of CLL. (e) The UMAPs showed the distribution of B cell subpopulation of each stage in CLL. (f) The violin plots present little expressed difference of different B cell markers in the 3 stages.

## Data Availability

The data used to support the findings of this study are included within the article.
